# The Application of the Big Data Medical Imaging System in Improving the Medical and Health Examination

**DOI:** 10.1155/2021/8251702

**Published:** 2021-09-16

**Authors:** Xiaojuan Zhou, Wenjun Ouyang

**Affiliations:** ^1^Henan Vocational College of Economics and Trade, Zhengzhou 450018, Henan, China; ^2^School of Economics and Management, China University of Geosciences (Wuhan), Wuhan 430000, China

## Abstract

To explore the application effect of the big data medical imaging tertiary diagnostic system in improving the medical and health examination, cases in township health centers were collected by the medical imaging tertiary diagnosis system. Clinical cases examined by the tertiary diagnostic system of big data medical imaging will be set as the observation group. Clinical cases not involved in the tertiary diagnostic system of big data medical imaging were set as the control group. The qualified rate, film positive rate, and film diagnosis accuracy between the two groups are compared, and X-ray perspective, X-ray examination, and CT multiple medical imaging examinations are used in two groups. The experimental results showed that the pass rate was 86.57%, positive rate was 72.32%, and diagnosis rate was 80.17%. Pass rate, positive rate, and diagnostic accuracy were higher than the control group (*P* < 0.05). X-line film is the most cost effective. CT examination has a high diagnostic sensitivity and can achieve a clear diagnosis of the benign and malignant diseases. The three-level diagnosis system of medical imaging has significantly improved and improved the technical level in the medical and health examination, which has good practical value.

## 1. Introduction

China's medical resources are relatively lacking and highly unbalanced in distribution. With the accelerating aging process in China, the contradiction between high-quality medical resources and the people's ever-improving demand for health services is becoming more and more serious [1]. Regional sharing of medical image information is the key to solve this problem. At present, with the implementation of China's “Internet +” development strategy and the active promotion of medical reform on hierarchical diagnosis and treatment and medical consociation construction, many places in China are trying to conduct regional PACS [2]. Medical imaging software, diagnostic medical imaging software, is suitable for almost all types of images. It can diagnose computer X-ray, digital photography, active imaging radiography, angiography, ultrasound, nuclear medicine, endoscopy, and ophthalmic diseases [3]. It can help doctors view 3D images and combine them with other images to get more information about the diagnosis. Godinho et al. found in their 2012 investigation that, in processing CT scan images of stroke patients, radiologists using the ResolutionMD mobile terminal can improve the speed by 24% compared with the PACS workstation, saving one patient every 11 minutes on average [4]. Kong and Chen estimated that the gap of talents in relevant majors in China in the next five years would be as high as 1.3 million; especially, big data talents with solid theoretical foundation and business practice experience across biomedical science and information science are in great shortage [5]. Zhou et al. believed that the future development of teleradiology would be more important [6]. On the basis of the present research, this paper expounds the characteristics of several radiological examinations commonly used in health examination in order to make reasonable application of this kind of examination. Specific x-ray fluoroscopy, health examination, X-ray, and multiple medical imaging tests are involved in the physical examination program. Through discussion and comparison, it is concluded that the X-ray film is the first choice and the most cost-effective method for screening chest diseases in the routine physical examination of most people at present. Ultrasound shows a high diagnostic sensitivity and can make a clear diagnosis of benign and malignant diseases [7, 8].

## 2. Materials and Methods

### 2.1. Clinical Data

The patients received imaging health examination in the mobile health center and were set as the control group. There were 2316 cases in the observation group, including 1169 males and 1147 females, aged from 2 to 83 years, with an average age of 55 ± 16.9 years. In the control group, there were 1,982 cases, including 1006 males and 976 females, ranging in age from 1 to 81 years, with an average age of 52 ± 18.3 years. There was no significant difference in age and gender between the two groups (*P* ≥ 0.05).

### 2.2. Research Methods

Doctors will upload the image data to the medical image level-3 diagnosis platform, so county hospital diagnostic center doctors can receive mobile phone SMS alerts and receive township hospital patients examination data. Doctors in the diagnostic center of county hospital can read diagnosis online, review, and issue diagnosis report and reply with electronic signature. Township health work site timely obtains and prints diagnostic reports to patients. For difficult cases, township doctors can upload the examination data to the central hospital for imaging consultation and generally complete the diagnosis or consultation within 1 hour [9].

### 2.3. Statistical Analysis

Data analysis was performed using SPSS 13.0. The measurement data are represented by mean ± standard difference (*x* ± *s*), compared using the *t*-test and *χ*^2^ test, and *P* < 0.05 is of statistical significance.

## 3. Results and Discussion

Among 2316 cases in the observation group, 2005 cases were qualified and 311 cases were unqualified, with a pass rate of 86.57%. In the control group of 1982 cases, 1391 cases were qualified and 591 cases were unqualified, with a qualified rate of 70.18%. The difference was statistically significant (*P* < 0.05), as shown in Table 1.

The main factors for unqualified cases are unphotographed positive position (32.13%), uploaded image quality defects (exposure, artifacts, and poor image quality) (28.58%), unmarked image left and right parts (25.12%), and failure to provide a complete medical history (14.17%).

In the observation group, 1675 cases were positive and 641 cases were negative, and the positive rate was 72.32%, while in the control group, 1167 cases were positive and 815 cases were negative, and the positive rate was 58.88%, among the 2316 cases. The difference was statistically significant (*P* < 0.05), as shown in Table 2.

The use of the medical imaging system for sentinel lymph nodes in the treatment of breast cancer is characterized by the ability to detect sentinel lymph node metastasis through some diagnostic methods. At present, the main methods for the clinical diagnosis of sentinel lymph node micrometastasis include continuous section, immunohistochemistry, and biopsy. However, in the actual operation process of the former two methods, all lymph nodes of patients need to be tested, which is a heavy workload and has great limitations in practical use; it is difficult to achieve the purpose of detection, so sentinel lymph node biopsy for breast cancer has become a widely used means in clinics. However, with the continuous development of medical technology, some scholars have proposed that colour ultrasound has a good effect on the diagnosis of sentinel lymph node micrometastasis [10].

Sixty cases of breast cancer patients admitted to a hospital from December 2014 to December 2015 were randomly selected as the research objects. All the selected patients were female, aged from 21 to 68 years, with an average age of 50.6 ± 5.7 years. Sites: 33 on the right side and 27 on the left side; there were 22 cases of invasive ductal carcinoma, 7 cases of mucinous adenocarcinoma, 8 cases of invasive lobular carcinoma, 10 cases of papillary adenocarcinoma, and 13 cases of medullary carcinoma. According to TNM stage T1-2N0M0, 25 cases were of the T1 stage (tumor diameter: <2 cm), 35 cases were of the T2 stage (tumor diameter: 2–5 cm), as shown in Table 3.

According to the material of the X-ray bulb tube anode, there are tungsten target and rhodium target. At present, molybdenum target is more commonly used for X-ray photography, which is of great value for the examination of breast cancer, the classic textbook description of the X-ray signs of breast cancer typically involves lesions that have formed masses or prominent nodules, with the improvement of people's health awareness and the popularization of medical knowledge, and the typical breast cancer is rarely found in the health examination; however, mammography is more difficult to diagnose early breast cancer with no history, no symptoms, no signs, and lesions of less than a certain volume than breast cancer with a history, symptoms, signs, and lesions of a certain volume; it depends even more on the personal experience of the diagnostician and the thinking environment at the time of reading the film, especially in women of reproductive age whose breast tissue has not degenerated; the value of mammography may be higher for those who have already been examined or self-examined by a doctor, especially for those who have been found to have suspicious nodules by ultrasound. Molybdenum target mammography of the breast generally takes a total of four films for the comparison between the upper and lower positions of both sides of the breast and the internal and external oblique positions, and the total amount of X-ray radiation cannot be ignored. Therefore, the indications for mammography should be mastered from the aspects of family history, age, medical history of the present illness, marriage, and child history to prevent the abuse from causing harm to women [11]. Some foreign anthologies suggest annual mammography and MRI examination for high-risk groups, and Liu Peifang also advocates MRI participation in the census of high-risk groups in China. Regular screening for breast cancer is necessary for high-risk groups. If mammography has the most comprehensive advantages compared with MRJ and ultrasound, another method of screening for breast cancer, it is worthwhile to make mammography the preferred method for early breast cancer screening in high-risk groups.

Due to the popularity of CT, in routine physical examination, further CT examination of lesions of solid organs in the digestive system, urogenital system, and other systems found by ultrasound examination and lung lesions found by the chest X-ray film can be used to differentiate benign from malignant lesions or evaluate their functions: patients with special indications of biochemical examination results can be screened for diseases of related organs: for patients with frequent dizziness and headache, in order to exclude cerebrovascular lesions, head CT can be included in the physical examination items if conditions permit; as a routine test, because of the high dose of X-ray radiation, how to use this new technique to maximize the diagnostic effect and accord with the principle of X-ray examination optimization is a subject worth studying. So, people tend to use low-dose spiral CT scans to screen for early lung cancer, and because of the low dose X-ray scans in low dose spiral CT scans, the thin-layer reconstruction technique is used instead of the thin-layer scan so that the dose of iatrogenic X-ray radiation of the subject is greatly reduced, and because the low-dose spiral CT scan requires less X-ray dose, the thermal effect of the CT tube is reduced, the loss of the CT tube is correspondingly reduced, the life of the tube is prolonged, and it is possible to reduce the charge reasonably. In addition, CD is used instead of film, which further saves the cost and makes it possible to charge the same fee for the low-dose spiral CT scan and chest CR and DR examination, which is easy to be accepted by people. For patients with cardiac symptoms, CT coronary imaging is undoubtedly necessary, but this examination can increase the amount of X-ray radiation in the subject, and the screening for coronary artery disease in the routine physical examination is still under study and questionable; some occupations have special physical requirements for practitioners. After a certain age, CT coronary imaging can be performed to screen for coronary artery lesions. In any case, you should respect the advice of your doctor as to whether or not to have a CT scan on a healthy subject, and you should never ask for a CT scan unless recommended by your doctor.

A total of 150 patients (55 males and 95 females) underwent thyroid nodule examination. The average age was 45.39 ± 5.96 years from 19 to 75 years. For all physical examination personnel, colour Doppler ultrasound was selected to carry out thyroid nodule disease diagnosis. The frequency of the ultrasonic probe was adjusted from 7.5 to 12 MHz such as Table 4.

Patients with hyperplasia of thyroid tissue are more likely to present with thyroid nodules. If the nature of the thyroid nodule is different, different clinical intervention measures should be selected [12]. For patients with benign thyroid nodule, conservative treatment and follow-up observation were mainly selected clinically. For physical examination personnel in the implementation of the thyroid nodule diagnosis process, the method of ultrasound examination is chosen, showing a high diagnostic sensitivity, and can be a clear diagnosis of benign and malignant diseases so as to ensure the smooth implementation of clinical effective thyroid nodule treatment methods.

As shown in Table 5, in the observation group of 2316 cases, 2213 cases were clearly diagnosed, 103 cases were undiagnosed, and the diagnosis rate was 95.55%. In the control group, 1589 cases were definitely diagnosed, 384 cases were undiagnosed, and the diagnosis rate was 80.17%. The difference was statistically significant (*P* < 0.05).

## 4. Conclusions

This paper discusses the application of several radiological images in normal physical examination. X-ray fluoroscopy; X-ray photography; color Doppler imaging; X-ray radiography has developed from screen radiography to computer radiography (CR) and the latest digital X-ray radiography (DR). Through the comparison of the positive rate of radiography in the observation group of 2316 cases, 1675 cases were positive and 641 cases were negative, and the positive rate was 72.32%, while in the control group of 1982 cases, 1167 cases were positive and 815 cases were negative, and the positive rate was 58.88%. Thus, this demonstrates that X-rays are the preferred and most cost-effective method of screening for chest disease during routine physical examinations. The choice of the ultrasound examination method shows a high diagnostic sensitivity, and the benign and malignant disease can be clearly diagnosed so as to ensure the successful implementation of the clinical effective treatment of thyroid nodules. The development of information technology has indeed provided us with great convenience and also promoted the development of medical imaging, teaching, and scientific research. It is combined with biotechnology, genetic engineering, and medical engineering. Hospitals at all levels should improve the understanding of digital large imaging, update their ideas, actively promote its application in hospitals, and strengthen personnel training. The rapid development of video technology has promoted the explosive coverage of video visual culture in today's society. When video visual culture enters the field of education, it will have a huge impact on the educational mode.

## Figures and Tables

**Table 1:** Comparison of imaging quality between the observation group and the control group.

Group	Qualified	Unqualified	Percentage of pass
Observation group (*n* = 2316)	2005	311	86.57
Control group (*n* = 1983)	1391	591	70.18

**Table 2:** Comparison of the positive rate of radiography between the observation group and the control group.

Group	Positive	Negative	Positive rate
Observation group (*n* = 2316)	1675	641	72.32
Control group (*n* = 1982)	1167	815	58.88

**Table 3:** Colour ultrasound results of breast cancer patients.

Position and type	This is an infiltrating ductal carcinoma	Mucous adenocarcinoma	This is an invasive lobular carcinoma	Papillary adenocarcinoma	Medullary carcinoma
On the right side	10	3	4	3	5
On the left side	12	4	4	7	8

**Table 4:** CT examination data of thyroid cancer patients.

	The number of people	Age	You have thyroid nodules	Thyroid cancer	Papillary carcinoma of the thyroid	Medullary thyroid carcinoma
Man	50	40–50	16	3	2	0
Woman	95	19–75	45	6	5	1

**Table 5:** Comparison of diagnostic rates between observation and control imaging subjects.

Group	Clarify a diagnosis	No clear diagnosis	Positive rate (%)
Observation group (*n* = 2316)	2213	103	95.55
Control group (*n* = 1982)	1589	384	80.17

## Data Availability

The data used to support the findings of this study are available from the corresponding author upon request.
